# Dynamic Evaluation of Transformation Ability for Emergency Scientific Research Achievements Based on an Improved Minimum Distance-Maximum Entropy Combination Weighting Method: A Case Study of COVID-19 Epidemic Data

**DOI:** 10.1155/2022/8005249

**Published:** 2022-08-12

**Authors:** Qingmei Tan, Juan Hui

**Affiliations:** College of Economics and Management, Nanjing University of Aeronautics and Astronautics, Nanjing, Jiangsu 211106, China

## Abstract

In the process of responding to major public health emergencies, the transformation of emergency scientific research results often faces many unfavourable factors such as limited resources, tight time, changes in needs, and lack of results. It is necessary to evaluate and analyze the ability to transform emergency scientific research results under public health emergencies, so as to rationally allocate emergency scientific research resources between subjects and regions, improve the efficiency of emergency results transformation, enhance emergency scientific research capabilities, and efficiently support incident prevention, control, and treatment. Starting from the patent level, this paper constructs an indicator system to evaluate the transformation ability of emergency scientific research results under major public health emergencies. It improves the minimum distance-maximum entropy combination weighting method to realize the static evaluation of transformation ability for emergency scientific research results from the perspective of patents, then constructs the dynamic evaluation model of transformation ability for emergency scientific research results in public health emergencies from the perspective of patents, and carries out the dynamic evaluation of the emergency scientific research achievements transformation ability of different subjects and different regions. We also improve the ER index, measure the static polarization effect of the transformation ability for regional emergency scientific research results, and consider the time factor to construct a dynamic polarization effect measurement model for the transformation ability of emergency scientific research achievement. Furthermore, this paper improves the measurement model of contribution degree to the polarization effect, and analyzes the contribution degree to polarization of the transformation ability for regional emergency scientific research results.

## 1. Introduction

Since the 21st century, public emergencies have occurred from time to time around the world, and the urgency and uncertainty of major public emergencies have posed a great challenge to global economic development. The sudden outbreak of the “COVID-19” epidemic in 2020 has had a great impact on the economic development of various countries and even the world, which is considered to be one of the greatest challenges and tragedies of the century after World War II [1]. It has resulted in the death of hundreds of thousands of people around the world, posed an urgent challenge to medical professionals, and exposed the weaknesses of national health systems [2, 3]. COVID-19 rapidly caused major economic and social disruptions on an unprecedented scale [4, 5].

Under the background of the above events, it is crucial to efficiently play the supporting role of scientific research results in the process of emergency management. However, the result transformation of emergency scientific research during the process of public health emergency response is often faced with many unfavourable factors such as limited resources, time constraints, and changing needs [6]. There is a great lack of scientific research results that can meet the emergency needs of health emergencies, and the update rate is fast. Therefore, it is of great significance to form a strong capacity to transform emergency scientific research results. It is beneficial to enhance the efficiency of emergency scientific research resources allocation among subjects and regions, strengthen the strength of emergency scientific research under emergencies, improve the efficiency of emergency results transformation, and provide scientific, safe, and effective emergency results guarantee for responding to public emergencies, so as to efficiently support the prevention, control, and treatment of events.

The transformation of scientific and technological achievements is a complex project, which is the key to the deep integration of scientific & technological innovation and economic development [7, 8]. In-depth studies have been conducted in the existing literature on the emergency scientific research system and its achievement transformation mechanism, the rapid response mechanism of emergency R&D, and the collaborative integration process and corresponding methods of emergency scientific research, which have laid a solid theoretical foundation for subsequent studies. However, there is a lack of empirical studies related to the transformation of emergency scientific research results in the existing literature, and no empirical analysis of the transformation capacity of emergency scientific research results and its spatial distribution characteristics under emergencies has been conducted. In addition, the evaluation of achievement transformation capability belongs to the multi-criteria decision-making problem. Due to many index attributes, insufficient index data and various evaluation methods, it is often difficult to accurately measure the science and technology achievements transformation ability, and a systematic, standard, and comprehensive evaluation model of achievement transformation ability has not been formed, and the influence of the time factor is mostly not considered. In the above research context, it is necessary to evaluate and analyze the transformation capacity of emergency scientific research results under public health emergencies. On the one hand, it is beneficial to enrich the theoretical achievements related to emergency scientific research management, provide the evaluation index system and transformation ability evaluation model of emergency scientific research results, and provide theoretical support for improving the transformation ability of emergency scientific research results under public health emergencies. On the other hand, it is conducive to clarifying the objective status of the transformation capacity of emergency scientific research results under public health emergencies, specifying the characteristics and differences of the transformation capacity of emergency results of different subjects and regions, clarifying the spatial distribution characteristics of the transformation of regional emergency results, and providing a realistic basis for improving the transformation capacity of emergency scientific research results under public health emergencies.

As one of the core measures of innovation output, patents are effective carriers of science and technology innovation information, which are more accurate, informative, and forward-looking than journal literature. Patents often contain huge technical and commercial values. According to the statistics of the World Intellectual Property Organization, 80% of global inventions and technical knowledge can be traced back to patent literature, and more than 90% of the world's innovation information originates from patents [9, 10]. In recent years, more and more experts and scholars have analyzed the capacity, efficiency, and status of scientific and technological innovation and transformation based on patent indicators and data.

To sum up, from the perspective of the patent, the indicator system to evaluate the transformation ability of emergency scientific research results under major public health emergencies is constructed. Using the G1 method, deviation maximization method, index difficulty weighting method, and CRITIC weighting method, the minimum distance-maximum entropy combined weighting method is improved to achieve the static evaluation of transformation ability of emergency scientific research achievements for each subject and each region. Then, a dynamic evaluation model of the transformation ability of emergency scientific research achievements under public health emergencies is constructed, and the transformation ability of emergency scientific research achievements for different subjects and regions is dynamically evaluated.

Combined with the characteristics of data and index, this paper improves the ER index to measure the static polarization effect of regional emergency scientific research achievement transformation ability. On this basis, considering the influence of event development time, the dynamic polarization effect measurement model of the transformation ability of emergency scientific research achievements is established. Furthermore, the existing measurement model of polarization contribution degree (it is abbreviated to PCD in this work) is improved to analyze the polarization effect contribution degree of transformation ability of emergency scientific research achievements in different regions.

In order to achieve the above research objectives, this paper is structured as follows(the frame structure diagram of this work is shown in Figure 1): Section 2 adopts the G1 method, deviation maximization method, index difficulty weight method, and CRITIC weight method to improve the minimum distance-maximum entropy combination weight method; based on this, static evaluation and dynamic evaluation models of the transformation ability of emergency scientific research achievements in the context of public health emergencies are constructed; the static polarization effect and dynamic polarization effect of transformation ability of emergency scientific research achievement in each region are calculated by improving ER index. Furthermore, it improves the measurement model of contribution degree to polarization effect.  Section 3 selects the number of valid invention patents (*X*1), patent maintenance period (*X*2), and the number of patent claims (*X*3) of emergency scientific research results under public health emergencies to construct an evaluation indicator system for the transformation ability of emergency scientific research results from the patent perspective.  Section 4 carries out static evaluation and dynamic evaluation for the transformation ability of emergency scientific research achievements under public health emergencies in China from the perspective of subject difference and regional difference. Based on this, the improved polarization effect index measurement model is used to analyze the polarization effect of the transformation ability of emergency achievements in the national and eight comprehensive economic zones; furthermore, the improved measurement model of PCD is applied to analyze the polarization effect contribution of the transformation ability of emergency scientific research achievements in different regions. Finally, Section 5 presents the important findings, limitations, and possible future research directions.

## 2. Evaluation Model

The existing literature mostly uses the combined subjective-objective weighting method to avoid the defects of subjective and objective weighting methods, to take into account the advantages of both methods, so as to improve the rationality, accuracy, and credibility of evaluation results. The minimum distance-maximum entropy combination weighting method integrates the two factors of “distance” and “entropy” to calculate the combined weights of subjective and objective multiple weighting methods [11].

The reason for applying the combined subjective-objective weighting method in this work mainly includes the following two aspects: (1) The combined subjective-objective weighting method can take into account the advantages of both subjective and objective weighting methods, and avoid the disadvantages of both methods [12, 13]. According to their experience and knowledge, the experts rank the importance of the evaluation indexes and assign the subjective weight. This method reflects the subjective will of the experts on the importance of the evaluation indexes, and the weight obtained is highly interpretable. However, the subjective weight cannot reflect the data information of the evaluation index, and the decision or evaluation results have strong subjective arbitrariness with poor objectivity, which also increases the burden on the decision analysts. The objective weight reflects the data information of the evaluation index and determines the weight mainly according to the relationship between the original data. It does not depend on subjective judgment of people and does not increase the burden of decision analysts. The decision-making or evaluation results have a solid mathematical theoretical basis. However, it will change with the change of the evaluation object set, that is, the stability is weaker than the subjective weight. It cannot reflect the importance of decision-makers to different indicators. At the same time, the objective weight cannot reflect the importance of the evaluation index itself, and is less explanatory than the subjective weight. The combined subjective-objective weighting method embodies the thought of system analysis. The combined subjective-objective weighting method can take into account the preference of decision-makers for evaluation indicators, and at the same time, reduce the subjective arbitrariness of weight assignment effectively, so as to achieve the unity of subjective and objective weight assignment of indicators, and make the evaluation results more accurate and reliable. (2) There is a lack of data related to the transformation of emergency scientific research achievements, and the evaluation indicators are limited. In this context, if only the subjective weighting method is used for evaluation, the index weight is greatly affected by the subjective preference of the evaluators, which will seriously reduce the rationality, accuracy, and credibility of evaluation results. To sum up, this work uses the combined subjective-objective weighting method to avoid the defects of subjective and objective weighting methods, to take into account the advantages of both methods, so as to improve the rationality, accuracy, and credibility of evaluation results.

Above all, on the basis of the existing literature, the minimum distance-maximum entropy combination weighting method is improved by applying the G1 method, deviation maximization method, index difficulty weighting method, and CRITIC weighting method, so as to achieve the static evaluation of the transformation ability of emergency scientific research achievements. Furthermore, a dynamic evaluation model of the transformation ability of emergency scientific research achievements under the background of public health emergencies is constructed.

### 2.1. Static Evaluation

The target standardization method is selected to normalize the original data of each index without dimensions. The calculation formula is as follows:

(1) $$\begin{array}{c} x_{ij}^{*}=\left\{\begin{array}{cc} \frac{x_{ij}}{x_{0j}}, & x_{ij}\text{is the positive index,}\\ \frac{x_{0j}}{x_{ij}}, & x_{ij}\text{is the negative index,}\\ \frac{1}{1+\left|x_{ij}-x_{0j}\right|}, & x_{ij}\text{is the moderate index,} \end{array}\right) \end{array}$$

where *x*_*ij*_ is the original data of the index, *x*_*ij*_^*∗*^ is the index data after dimensionless processing, *x*_0*j*_ is the ideal value of the *j*th indicator, *i* is the ordinal number of the evaluation objects (*i*=1,2,…, *n*) , and *j* is the ordinal number of the evaluation indicators (*j*=1,2,…, *m*).

#### 2.1.1. G1 Method

As an efficient method for subjective assignment of indicators, the G1 method determines the relationship between the importance of indicators based on the sequential relationship between indicators, and then determines the G1 subjective weight of each indicator. This method facilitates the integration of the rich theoretical and practical experience of assessment experts [14]. The main steps are as follows:

(a) The experts rank the indicators *x*_*j*_ according to their importance, satisfying *x*_1_ ≥ *x*_2_ ≥ ⋯≥*x*_*m*_ (*j*=1,2,…, *m*).
(b) Calculate the importance ratio *r*_*k*_(*k*=*m*, *m* − 1,…, 3,2) between adjacent indicators, i.e., the ratio of the relative importance degree of indicators *x*_(*k* − 1)_ and *x*_*k*_. The reference for the assignment of *r*_*k*_ is listed in Table 1.
(c) Obtain the weight of the last indicator *x*_*m*_.
  (2) $$\begin{array}{c} w_{m}={\left(1+\sum_{i=2}^{m}\prod_{k=i}^{m}r_{k}\right)}^{-1}. \end{array}$$
(d) Calculate the weights of other indicators in reverse order,
  (3) $$\begin{array}{c} w_{\left(k-1\right)}=w_{k}\cdot r_{k}\left(k=m,m-1,\ldots ,3,2\right). \end{array}$$

Finally, the subjective weighting of indicators is realized and the subjective weight [*w*_1_, *w*_2_,…, *w*_*m*_] of each indicator by G1 method is obtained..

#### 2.1.2. Deviation Maximization Method

The deviation maximization method is based on the statistical distribution characteristics of the specific data of the evaluation indexes, and the objective weighting of the indexes is achieved based on the difference between the data of each evaluation object under different indexes [15]. It is considered that the greater the difference between different data of an indicator, the more significant the impact of the indicator on the final evaluation results and the greater its weight. The calculation process is as follows:

(a) The deviation between the evaluation object *M*_*i*_ and other evaluation object *M*_*j*_ is denoted by *Q*_*ij*_(*w*) ,
  (4) $$\begin{array}{c} Q_{ij}\left(w\right)=\sum_{r=1}^{n}\left|x_{ij}^{*}\cdot w_{j}-x_{rj}^{*}\cdot w_{j}\right|\\ =w_{j}\cdot \sum_{r=1}^{n}\left|x_{ij}^{*}-x_{rj}^{*}\right|,\;r=1,2,\cdots ,n, \end{array}$$
where, *x*_*ij*_^*∗*^ is the index data value after dimensionless processing.
(b) Let *Q*_*j*_(*w*) be the total deviation of all evaluation objects from other objects under the *j*th index,
  (5) $$\begin{array}{c} Q_{j}\left(w\right)=\sum_{i=1}^{n}Q_{ij}\left(w\right)\\ =w_{j}\cdot \sum_{i=1}^{n}\sum_{r=1}^{n}\left|x_{ij}^{*}-x_{rj}^{*}\right|. \end{array}$$
Constructing and solving the following optimization model on the basis of the deviation maximization principle,
  (6) $$\begin{array}{c} \max Q\left(w\right)=w_{j}\cdot \sum_{j=1}^{m}\sum_{i=1}^{n}\sum_{r=1}^{n}\left|x_{ij}^{*}-x_{rj}^{*}\right|\\ s.t.\left\{\begin{array}{cc} \sum_{j=1}^{m}w_{j}^{2} & =\;1.\\ w_{j} & \geq \;0. \end{array}\right) \end{array}$$
(c) The optimal solution of the optimization model (6) is normalized to obtain the weights of each index,
  (7) $$\begin{array}{c} w_{j}=\frac{\sum_{i=1}^{n}\sum_{r=1}^{n}\left|x_{ij}^{*}-x_{rj}^{*}\right|}{\sum_{j=1}^{m}\sum_{i=1}^{n}\sum_{r=1}^{n}\left|x_{ij}^{*}-x_{rj}^{*}\right|}. \end{array}$$

#### 2.1.3. Indicator Difficulty Weighting Method

The indicator difficulty weighting method completes objective evaluation based on the growth difficulty of evaluation indicators, and analyzes the growth difficulty of indicators according to the deviation degree between the maximum value and the mean value of indicator data, so as to ensure that the evaluation results do not lose balance due to the skewing of evaluation objects toward the large weighted indicators [16]. Evaluation indicators with greater growth difficulty usually have greater differentiation, and their weights can enhance the final evaluation result differentiation when they are larger. The weighting steps are as follows:

(a) Calculate the deviation degree *z*_*j*_ between the maximum value and the mean value of the *j* th evaluation index data,
  (8) $$\begin{array}{c} z_{j}=\frac{\max_{i}\left(x_{ij}^{*}\right)-\bar{x_{j}^{*}}}{\sigma_{j}}. \end{array}$$
(b) Obtain the objective weight *w*_*j*_ of the *j*th evaluation indicator under the indicator difficulty weighting method,
  (9) $$\begin{array}{c} w_{j}=\frac{z_{j}}{\sum_{j=1}^{m}z_{j}}. \end{array}$$

#### 2.1.4. CRITIC Method

The CRITIC indicator weighting method calculates the objective weight of each indicator based on “contrast strength” and “conflict” [14, 17]. Among them, the “contrast strength” between indicators can be calculated by the standard deviation of indicators, and the “conflict” is mostly reflected by the correlation between indicators. This method is widely used in decision-making problems in many fields such as economics, management, information, and so on. The weighting procedure is as follows:

(a) Calculate the correlation coefficient *r*_*jj*′_ of the *j*(*j*=1,2,…, *m*)th indicator with other indicators based on dimensionless processing of data values,
  (10) $$\begin{array}{c} r_{jj^{\prime }}=\frac{1/n-1\sum_{i=1}^{n}\left(y_{ij}-{\bar{y}}_{\cdot j}\right)\left(y_{ij^{\prime }}-{\bar{y}}_{j^{\prime }}\right)}{\sigma_{j}\sigma_{j^{\prime }}}, \end{array}$$
where, ${\bar{y}}_{j}$ is the mean value of the *j*th index and *σ*_*j*_ is the standard deviation of the *j*th index.
(b) Obtain the total conflict *f*_*j*_ of the *j*th index,
  (11) $$\begin{array}{c} f_{j}=\sum_{j^{\prime }=1}^{m}\left(1-r_{jj^{\prime }}\right). \end{array}$$
(c) Calculate the amount of information *c*_*j*_ for the *j*th indicator.
  (12) $$\begin{array}{c} c_{j}=\sigma_{j}f_{j}. \end{array}$$
(d) Obtain the weight *w*_*j*_ of the *j*th index under the CRITIC weighting method,
  (13) $$\begin{array}{c} w_{j}=\frac{c_{j}}{\sum_{j=1}^{m}c_{j}}. \end{array}$$

#### 2.1.5. Improved Combination Weighting Method with Minimum Distance-Maximum Entropy

The weights *w*_*j*_^(*q*)^(*q*=1,2,3,4) are obtained by combining the G1 method, the deviation maximization method, the indicator difficulty weighting method, and the CRITIC weighting method, respectively. Based on the existing literature [11], the improved combined weights are obtained as

(14) $$\begin{array}{c} w_{j}=\sum_{q=1}^{4}\lambda_{q}w_{j}^{\left(q\right)}, \end{array}$$

where *λ*_*q*_ denotes the weight combination coefficient (∑_*q*=1_^4^*λ*_*q*_=1), and *w*_*j*_^(*q*)^ denotes the weight of the *j*th indicator obtained by the *q*th weighting method. The combination coefficient *λ*_*q*_ is determined by considering the factors of “distance” and “entropy value” [18–20].

(a) Take the minimum value of the generalized distance between weighted values of different evaluative objects and the ideal point,
  (15) $$\begin{array}{c} \text{min}\sum_{i=1}^{n}d_{i}=\sum_{i=1}^{n}\sum_{j=1}^{m}\sum_{q=1}^{4}\lambda_{q}w_{j}^{\left(q\right)}\left(1-x_{ij}^{*}\right). \end{array}$$
(b) The “maximum entropy” principle is applied to prevent individual weighting methods from being removed due to their little impact on the combined assignment results. The following objective function is constructed based on the principle of “consistency maximization” of the weight assignment results,
  (16) $$\begin{array}{c} \text{max}H=-\sum_{q=1}^{4}\lambda_{q}\text{ln}\lambda_{q}. \end{array}$$
Considering the above objectives together, the model is constructed:
  (17) $$\begin{array}{c} \text{min}\left[\mu \sum_{i=1}^{n}\sum_{j=1}^{m}\sum_{q=1}^{4}\lambda_{q}w_{j}^{\left(q\right)}\left(1-x_{ij}^{*}\right)+\left(1-\mu \right)\sum_{q=1}^{4}\lambda_{q}\text{ln}\lambda_{q}\right]\\ s.t.\left\{\begin{array}{cc} \sum_{q=1}^{4}\lambda_{q} & =\;1,\\ \lambda_{q} & \geq \;0, \end{array}\right) \end{array}$$
where the parameter 0〈*μ*〈1 represents the balance coefficient between the two objectives (distance minimization, entropy maximization), usually taken as *μ*=0.5, and *x*_*ij*_^*∗*^ is the data value after dimensionless process of the index.
(c) By solving model (17), the optimal solution *λ*_*q*_ of the weight combination coefficients is obtained. The solved *λ*_*q*_ is substituted into equation (14) to obtain the minimum distance-maximum entropy combination weight *w*_*j*_ for each evaluation index.

Furthermore, the static evaluation value *I*_*i*_ of the transformation ability of scientific research achievements under public health emergencies is calculated,

(18) $$\begin{array}{c} I_{i}=\sum_{j=1}^{m}w_{j}\cdot x_{ij},\;i=1,2,\cdots ,n. \end{array}$$

### 2.2. Dynamic Evaluation

The realization of dynamic comprehensive evaluation must first determine the time series weights [11, 21]. On the basis of static evaluation, the influence of time factors is emphasized, and the time-series weighted average operator is applied for secondary weighting, so as to achieve a comprehensive dynamic evaluation of each evaluation object in the time interval [1, *h*]. The main evaluation steps are as follows:.

(a) Obtain the static evaluation value *I*_*i*_(*t*) of the *i*th evaluated object at moment *t* based on the static evaluation model,
(b) Calculate the time series weights. Set the time series weight vector be *w*_*t*_ : *w*_*t*_=(*w*_1_, *w*_2_,…,*w*_*h*_)^*T*^, solve the model of the nonlinear programming problem below, and obtain *w*_*t*_,
  (19) $$\begin{array}{c} \max\left(-\sum_{t=1}^{h}w_{t}\text{ln}w_{t}\right)\\ s.t.\left\{\begin{array}{cc} \sum_{t=1}^{h}\left(h-t\right)/\left(h-1\right)w_{t} & =\;\theta ,\\ \sum_{t=1}^{h}w_{t} & =\;1, \end{array}\right) \end{array}$$
where the parameter *θ* is the importance degree of time, and its assignment values are listed in Table 2.
(c) Using the time-series weighted average operator, the static evaluation value *I*_*i*_(*t*) obtained from (18) is secondarily weighted to realize the dynamic comprehensive evaluation of the *i*th evaluation object,
  (20) $$\begin{array}{c} L_{i}=A\left(\langle 1,I_{i}\left(1\right)\rangle ,\langle 2,I_{i}\left(2\right)\rangle ,\cdots ,\langle h,I_{i}\left(h\right)\rangle \right)\\ =\sum_{t=1}^{h}I_{i}\left(t\right)\cdot w_{t}. \end{array}$$

### 2.3. Polarization Effect Model

The theory of polarization effect was first proposed by Perroux [22]. The most commonly used polarization effect indices in the existing literature are ER index, TW index, KZ index, and Wolfson index. Scholars use single polarization index or multi-polarization index to measure the level of regional polarization effect, and mostly use the above polarization indexes to analyze the spatial polarization effect in the fields of regional economic development, scientific and technological innovation, and industrial innovation, etc. At the same time, many research results show that under the influence of institutions and policies, science and technology innovation mostly presents spatially unbalanced development [23]. Theoretical models such as “growth poles,” “gradient shift,” and “core-edge” all emphasize the unbalanced allocation of scientific and technological innovation resources under the condition of limited resources. In the abovementioned research context, scholars have used the polarization effect model to analyze the spatial evolution characteristics of the regional innovation polarization effect.

#### 2.3.1. Improved ER Index

Based on the basic principle of ER index and referring to existing literature [24], the static polarization effect measurement model of transformation capability of regional emergency scientific research results is constructed, and the static polarization degree (it is abbreviated to SPD in this work) index of emergency scientific research results transformation capability *f*_*ER*_*S*_ is calculated,

(21) $$\begin{array}{c} f_{ER\_S}=A^{*}\sum_{i=1}^{n}\sum_{j=1}^{n}p_{i}^{1+\partial }p_{j}\left|I_{i}-I_{j}\right|, \end{array}$$

where *n* is the total number of evaluation objects in a region, i.e., the number of evaluated areas in a region; *p*_*i*_ and *p*_*j*_ are the proportion of a certain variable value (in the *i*th and *j*th area) in the whole country or the region, respectively. *A*^*∗*^ is the standardized coefficient of polarization effect index, *A*^*∗*^=1+2*μ*^1+*α*^ (where, *μ*=∑_*i*=1_^*n*^*p*_*i*_*I*_*i*_). Meanwhile, *α* ∈ [0,1.6], the value should be as large as possible, which is conducive for reflecting the polarization characteristics of the region, and usually takes *α*=1.5. Different from the original model, *I*_*i*_ and *I*_*j*_ are the static evaluation values of emergency scientific research results transformation ability in *i*th and *j*th areas within a certain region under a public health emergency, respectively.

#### 2.3.2. Dynamic Polarization Degree

Based on the static polarization index *f*_*ER*_*S*_ of the transformation capability of emergency scientific research achievements, considering the influence of time factors, the time-series weighted average operator is applied to realize the secondary weighting of *f*_*ER*_*S*_. The dynamic polarization effect measurement model of the transformation capability of emergency scientific research results during the time interval of [1, *h*] is constructed, and the dynamic polarization degree (which is abbreviated to DPD in this work) index *f*_*ER*_*D*_ of the transformation capability of regional emergency scientific research results is calculated,

(22) $$\begin{array}{c} f_{ER\_D}=A\left(\langle 1,f_{ER\_S}\left(1\right)\rangle ,\langle 2,f_{ER\_S}\left(2\right)\rangle ,\cdots ,\langle h,f_{ER\_S}\left(h\right)\rangle \right)=\sum_{t=1}^{h}f_{ER\_S}\left(t\right)\cdot w_{t}, \end{array}$$

where *f*_*ER*_*S*_(*t*) is the SPD index of emergency scientific research results transformation capability at moment *t*, *w*_*t*_ is the time series weight, and *t* ∈ [1, *h*].

#### 2.3.3. Polarization Contribution Degree

In the context of emergencies, the emergency scientific research resources are limited, the time is urgent, the demand is changeable, and the relevant evaluation index data of achievement transformation ability are limited. In order to further analyze the contribution of a certain area to the polarization effect of the transformation ability of emergency scientific research achievements in the region, on the basis of existing literature and combined with the characteristics of the evaluation index data of the transformation ability of emergency science research achievements, the measurement model of PCD is improved, so as to construct the measurement model of polarization contribution degree for the transformation ability of emergency science research results under public health emergencies, and calculate the polarization contribution *C*_*ERi*_ of the transformation ability of emergency scientific research achievements in *i* th area,

(23) $$\begin{array}{c} C_{ERi}=1-\frac{f_{ER\_D}^{\left(i\right)}}{f_{ER\_D}}, \end{array}$$

where *f*_*ER*_*D*_^(*i*)^ denotes the dynamic polarization degree index of a region without *i*th area, and *f*_*ER*_*D*_ denotes the dynamic polarization degree index of a region containing *i*th area. The PCD *C*_*ERi*_ is greater than 0, which indicates that there is a promoting effect of *i*th area on the polarization effect of emergency scientific research results transformation ability in the region; conversely, it produces an inhibiting effect.

## 3. An Evaluation Indicator System for the Emergency Scientific Research Results Transformation Ability from the Patent Perspective

The patent is an important carrier of achievement transformation and scientific research innovation, and an important indicator for judging the level of achievement transformation and the strength of scientific research innovation, which has an important impact on technology breakthroughs and innovation development. The number of patents and their changing trends often reflect the scientific research strength and innovation competitiveness of a country or region [25]. In recent years, patent data and information have become an important evaluation index for domestic and foreign experts and scholars to analyze the achievement transformation ability and innovation potential of scientific research. The U.S. “Bayh-Dole Act” promotes the achievement transformation in the form of patent law amendments, which also shows the particularity and importance of patent for the achievement transformation from the side [26]. Therefore, it is reasonable and feasible to analyze the ability, efficiency, and current situation of scientific & technological innovation and achievement transformation based on patent data.

In the context of major public health emergencies, the statistical caliber and cycle of monthly progress data in various regions are different. Some districts only publish quarterly data, not monthly progress data. Therefore, according to the principle of index system construction, “systematic, typical, dynamic, scientific, operable, and comprehensive,” applying with the “grounded theory” and Delphi method, the primary index set and the optimized index set are gradually obtained through the rigorous index system construction process. Then, combining the availability of progress data (monthly), the index set is revised and improved after discussion with experts and team members. Finally, the evaluation indicator system for the emergency scientific research results transformation ability from the patent perspective is constructed (as shown in Table 3). Due to the limited space, more specific construction process, selection basis, and connotation explanation of the index system can be obtained by contacting the author.

After a rigorous screening process of indicators, the number of valid invention patents (*X*1), patent maintenance period (*X*2), and number of patent claims (*X*3) of emergency scientific research results under public health emergencies are selected to construct an index system to evaluate the transformation ability of emergency science research results from the patent perspective, as shown in Table 3. Among them, the number of valid invention patents and the number of patent claims are both positive indicators, and the patent maintenance period is an adaptive indicator. Specifically, the number of valid invention patents is a key indicator reflecting the quality of patents and an important indicator measuring the contribution of industrial economy to employment; the patent maintenance period is one of the important indicators reflecting the operation effectiveness of the patent system and the advantages and disadvantages of the patent maintenance system, and is regarded as a key factor measuring the technical and economic value of patents; the number of patent claims is the core of patents and determines the protection scope of patent rights. Based on the above evaluative indicator system, the transformation ability of emergency science research results in public health emergencies is evaluated from the patent perspective.

## 4. Empirical Analysis

The static evaluation and dynamic evaluation of the transformation ability of emergency science research results under public health emergencies in China are conducted from two perspectives: subject differences and regional differences. From the perspective of subject differences, the transformation ability of emergency scientific research results of five major subjects–enterprise, institution (mainly hospital), individual, universities, and research institute–are evaluated. From the perspective of regional differences, the capacity of 31 provinces, municipalities, and autonomous regions in China are evaluated (Hong Kong, Macao, and Taiwan are not evaluated for the time being due to insufficient data); based on this, the improved polarization effect index measurement model is used to analyze the polarization effect of the transformation ability of emergency achievements in the national and eight comprehensive economic zones; furthermore, the improved measurement model of PCD is applied to analyze the polarization effect contribution of the transformation ability of emergency scientific research achievements in different regions.

### 4.1. Data Sources

The empirical data originate from “Patyee” patent search database. The database is an authoritative search and analysis platform with independent intellectual property rights, which provide data services for government departments, universities, research institutes, and enterprises all year round; the data are accurate, comprehensive, and timely updated. It covers more than 100 countries and regions, containing more than 140 million patent data. The search keywords are set to “COVID-19” or “Novel coronavirus,” the patent status is set to “valid,” and the time limit for patent disclosure is set from “March 2020” to “May 2021.” After filtering and collating, we obtained a total of 458 (for 15 months) valid patents related to “COVID-19” or “Novel coronavirus” from 31 provinces, municipalities, and autonomous regions in China.

### 4.2. Evaluation Results and Analysis

#### 4.2.1. Perspective of Subject Difference

*(1) Static Evaluation.*

Based on the improved minimum distance-maximum entropy combination weighting method, the combination weights *w*_*j*_(*j*=1,2,3) of the evaluation indexes *X*1–*X*3 for the transformation ability of emergency scientific research results in public health emergencies under the perspective of differences in scientific research subjects are calculated and shown in Table 4.

Based on equation (18), the static evaluation results of the transformation ability of emergency research results are obtained for each subject (from March 2020 to May 2021) under the background of “COVID-19” epidemic (shown in Table 5). In order to analyze the static evaluation results more visually and present the rules and differences, Figure 2 is drawn according to Table 5.

As can be analyzed from Table 5 and Figure 2, in the static evaluation of the transformation ability of emergency scientific research results of different scientific research subjects under the “COVID-19” epidemic, the average value of the transformation ability (from March 2020 to May 2021) ranks as follows: enterprise (0.920), institution (0.256), individual (0.158), university (0.152), and research institute (0.126). Among them, the transformation ability of enterprise emergency scientific research achievements is generally strong, far exceeding the average value of the same period, and the transformation power of achievements is lasting; transformation ability of emergency scientific research results of institution is lower than enterprise, close to the average value of the same period, with an overall “*W*”-type change trend; emergency scientific research results transformation ability of the individual, university, and research institute is close, lower than the average value of the same period. At the same time, enterprise, institution, and individual all demonstrated a strong transformation ability to emergency scientific research results at the early stage of the epidemic, providing strong scientific research results to support the epidemic response. In addition, enterprise is an important innovation subject in science and technology R&D, and hospital is an important scientific research subject in the clinical front line, both of which have a strong transformation ability of emergency scientific research results, The evaluation results are in line with objective facts, which proves the reasonableness, reliability, and scientificity of the evaluation model in this paper from the side.

*(2) Dynamic Evaluation*.

Based on the dynamic evaluation step (b), the time series weights *w*_*t*_(*t*=1,2,…, 15) are determined (as shown in Table 6). To highlight the importance of recent data, set *θ*=0.4.

Based on equation (20), the dynamic evaluation results of the transformation ability of emergency research results of each subject under the “COVID-19” epidemic are obtained (as shown in Table 7). The dynamic evaluation values of each indicator are also calculated (seen in Table 8). For visual analysis, Figure 3 is drawn.

As can be seen from Table 7, in the dynamic evaluation of the transformation ability of emergency scientific research achievements for each subject, enterprise has the strongest ability to transform emergency scientific research results and exceeds the average value; institution (mainly hospital) has weaker ability to transform emergency scientific research results than enterprises and is close to the average value; the transformation ability of emergency science research results of individual, university, and research institute is weaker and lower than the average value. As can be seen from Table 8 and Figure 3, enterprise ranks high in all aspects of the transformation of emergency achievements, and the advantage of patent maintenance period is more prominent; other subjects have smaller differences in the number of valid invention patents and claims, and the gap between their patent maintenance period and enterprise is larger.

#### 4.2.2. Perspective of Region Difference

*(1) Static Evaluation.*

Based on the improved minimum distance-maximum entropy combination weighting method, the combination weights *w*_*j*_(*j*=1,2,3) of the evaluation indexes *X*1–*X*3 for the transformation ability of emergency scientific research results in public health emergencies under the perspective of regional differences are calculated and shown in Table 9.

Based on equation (18), the static evaluation results of the transformation capacity of emergency research results by region and month are obtained under the “COVID-19” epidemic (as shown in Table 10). In order to analyze the static evaluation results more visually and present the rules and differences, Figure 4 is drawn according to Table 10.

As can be seen from Table 10 and Figure 4, the top 5 regions in the static evaluation of the transform ability of emergency scientific research achievements in different regions (from March 2020 to May 2021) under the “COVID-19” epidemic are Guangdong (0.673), Beijing (0.580), Jiangsu (0.541), Shanghai (0.272),and Tianjin (0.180). Among them, the transformation ability of emergency scientific research achievements of Guangdong is generally strong, exceeding the average value of the same period as a whole; Beijing is weaker than Guangdong, but still at a higher level and exceeds the mean value of the same period; Jiangsu exceeds the average value in the same period but fluctuates more obviously and shows a downward trend in the near future; Shanghai shows a significant upward trend in the near future and has outstanding development potential; Tianjin is lower than the average value of the same period, and the declining trend is more significant. Further analyze the transformation characteristics of emergency achievements for Guangdong, Beijing, and Jiangsu. Specifically enterprises and institutions in Guangdong have a large number of patents related to “COVID-19” with good quality; the transformation work of emergency scientific research results in Guangdong started quickly (after the outbreak of the epidemic, a strong transformation ability of emergency scientific research results is rapidly formed), and the advantages of emergency R&D is outstanding, the achievements of which are mostly concentrated in reagents (boxes), pharmaceutical compositions, epidemic prevention equipment, etc. Enterprises and institutions in Beijing also show strong advantages in emergency R&D, with achievements mostly concentrated in reagents (boxes), vaccines, and their preparation methods, peptides or their combinations for detecting (or inhibiting) viruses, etc. Enterprises and research institutes in Jiangsu are more prominent in emergency R&D, with results mostly focused on epidemic prevention equipment, reagents (boxes), interfering nucleic acids and their combinations, etc.

*(2) Dynamic Evaluation.*

According to the dynamic evaluation step (b), the time series weights *w*_*t*_(*t*=1,2, ⋯, 15) are determined by making *θ*=0.4, and the results are consistent with Table 6. Based on equation (20), the dynamic evaluation results of the transformation capacity of emergency scientific research results in each region under the “COVID-19” epidemic are obtained (as shown in Table 11). The dynamic evaluation values of each indicator are also calculated (As shown in Table 12.). For visual analysis, Figure 5 is drawn.

As can be seen from Table 11, the top 5 regions in the dynamic evaluation of the transformation ability of the emergency scientific research results are Guangdong (0.654), Beijing (0.651), Jiangsu (0.567), Shanghai (0.288), and Tianjin (0.178). Among them, Guangdong has the strongest ability to transform the emergency scientific research results, which is much larger than the average value; Beijing is second only to Guangdong in the transformation ability of the emergency scientific research achievements, which is also much larger than the average value. From Table 12 and Figure 5, it can be analyzed that Guangdong ranks first in the dynamic evaluation of all indicators of transformation of emergency achievements, the dynamic evaluation of each indicator exceeds its average value, and the advantages of the patent maintenance period and the number of claims for Guangdong are more prominent; Beijing ranks first in the dynamic evaluation of the number of valid invention patents, and its dynamic evaluation of other indicators also exceeds the average value; Jiangsu, Shanghai, and Tianjin are relatively consistent in the dynamic evaluation of each indicator, and Jiangsu has certain advantages in patent maintenance period. The dynamic evaluation of all indicators of Shanghai and Tianjin are lower than the average value.

*(3) Transformation Ability of Emergency Scientific Research Achievements in the Eight Comprehensive Economic Zones*.

For the analysis of spatial distribution characteristics of the transformation capability of emergency scientific research results more accurately, the average value of the static (dynamic) evaluation value of the transformation capability of emergency scientific research results in each province and city within each economic zone is taken as the static (dynamic) evaluation value of the transformation capability of emergency scientific research achievements in that economic zone (according to the principle of dividing eight comprehensive economic zones in China), as shown in Tables 13 and 14. From the table, it could be analyzed that, under the background of the “COVID-19” epidemic, the top 3 comprehensive economic zones in terms of dynamic evaluation of transformation ability of emergency scientific research results are the Eastern Coastal Economic Zone (0.322), Northern Coastal Economic Zone (0.237), and Southern Coastal Economic Zone (0.235), which have stronger transformation ability of emergency scientific research results; Middle Yellow River Economic Zone and Northwest Economic Zone have lower dynamic evaluation value of transformation ability of emergency scientific research results and weaker transformation ability of emergency scientific research results. In order to more intuitively analyze the static evaluation results of transformation ability of emergency scientific research results for each comprehensive economic zone, Figure 6 is drawn. It can be seen from this figure that the Eastern Coastal Economic Zone, Northern Coastal Economic Zone, and Southern Coastal Economic Zone maintain a high level of transformation ability of emergency scientific research results in each month from March 2020 to May 2021, which is consistent with the dynamic evaluation results. In conclusion, during the response to the “COVID-19” epidemic, the eight comprehensive economic zones have significant differences in the transformation capacity of emergency scientific research results and unbalanced spatial distribution.

*(4) Polarization Effect Analysis.*

Based on the static polarization effect measurement model (equation (21)), the SPD of transformation capability of emergency scientific research results in China is calculated; furthermore, according to equation (22), the dynamic polarization degree (which is abbreviated to DPD in this work) of emergency scientific research results in China is calculated, and the results are illustrated in Figure 7. The analysis shows that the SPD of transformation capability of emergency scientific research results in China fluctuates under the “COVID-19” epidemic, and the polarization level is low, indicating that the resource aggregation status of national emergency research is constantly adjusting with the epidemic development stage, and the resource aggregation process in the global scope has not yet shown the characteristics of order and large scale. The “polarization” and “diffusion” of transformation capability of emergency scientific research results in China are alternating, and the polarization effect is weak. In addition, the dynamic polarization level of transformation ability of emergency scientific research results in China is low, indicating that the transformation ability of emergency scientific research results at the national level does not form a significant polarization effect considering the influence of time factor.

Furthermore, the top 3 comprehensive economic zones in terms of the dynamic evaluation value of the transformation capacity of emergency scientific research results under the “COVID-19” epidemic are taken as the research objects to analyze their polarization effect of the transformation capacity of emergency scientific research results, as shown in Tables 13 and 14. It can be seen from the table that the static polarization level of the transformation capacity of emergency scientific research achievements in the Northern Coastal Economic Zone, Eastern Coastal Economic Zone, and Southern Coastal Economic Zone is significantly different, and the DPD is low; the static (dynamic) polarization effect of transformation ability of emergency scientific research results in the Southern Coastal Economic Zone is weaker. The results show that the above three comprehensive economic zones have not formed a more obvious and stable polarization effect of emergency scientific research results transformation ability; under the “COVID-19” epidemic, their resources gathering of emergency scientific research results transformation has not formed an orderly and large-scale development trend.

In order to more intuitively analyze the polarization effect of the top 3 comprehensive economic zones in terms of the transformation ability of emergency scientific research results, Figure 8 is drawn according to Table 14. It can be seen from the figure that under the “COVID-19” epidemic, the polarization effect of the transformation ability of emergency scientific research achievements in the above three comprehensive economic zones fluctuates obviously, and the polarization level is high in some months; the polarization level of the transformation capacity of emergency scientific research results in the Southern Coastal Economic Zone is low and the most unstable. The results show that the trend of resource aggregation of emergency research results transformation in the above three economic zones is unstable, and the “polarization” and “diffusion” effects of transformation ability of emergency research results occur alternately. This is consistent with the characteristics of emergency science research results transformation. Within the process of responding to major public health emergencies, due to multiple factors such as time urgency, limited resources, changing needs, and differences in the foundation, the trend of resource aggregation and capacity polarization of emergency scientific research results in each region is unstable, which are constantly adjusted and optimized with the development stage of the event. Through coordination and cooperation with surrounding areas, an efficient and stable transformation capacity of emergency scientific research achievements are gradually formed. This is a long-term process of continuous iteration and evolution.

Based on the conclusion of the above polarization degree analysis and on equation (23), the PCD of emergency scientific research results transformation capacity for each province and city within the three major economic zones of the Northern Coastal Economic Zone, Eastern Coastal Economic Zone, and Southern Coastal Economic Zone are calculated, as shown in Table 15. Specifically: (1) Within the Northern Coastal Economic Zone, the PCD of transformation capacity of emergency scientific research results in Tianjin is the largest; the PCD of Tianjin, Hebei, and Shandong are all greater than 0, which promote the polarization effect of transformation capacity of emergency scientific research results in the Northern Coastal Economic Zone. The PCD of Beijing is less than 0. Further analysis suggests that Beijing is the core city for dispatching emergency research resources in China, and its transformation ability of emergency scientific research results has a frequent “polarization” and “diffusion” effect on other regions, so it has an inhibiting effect on the polarization effect of emergency research results transformation capacity in the Northern Coastal Economic Zone, and its PCD is less than 0, which is reasonable. (2) Within the Eastern Coastal Economic Zone, the PCD of emergency scientific research results transformation capacity in Shanghai is the largest; the PCD of Shanghai, Jiangsu, and Zhejiang are all greater than 0, which all have the positive contribution to the polarization effect of transformation capacity of emergency scientific research results in the Eastern Coastal Economic Zone. (3) Within the Southern Coastal Economic Zone, the PCD of emergency scientific research results transformation ability in Guangdong is the largest; the PCD of Fujian, Guangdong, and Hainan are all greater than 0, which all promote the polarization effect of transformation ability of emergency scientific research results in the Southern Coastal Economic Zone.

## 5. Conclusion

The analysis of the transformation capacity of emergency scientific research results under public health emergencies is conducive for the reasonable allocation of inter-subject and inter-regional emergency scientific research resources, the improvement of the transformation efficiency of emergency results, and the enhancement of emergency scientific research strength, so as to efficiently support the prevention, control, and treatment of the event. Based on the improved minimum distance-maximum entropy combination weight, from the patent level, it carries out the static and dynamic evaluation for the transformation ability of emergency science research results of different subjects and different regions under major public health emergencies. Furthermore, the polarization effect model is improved, and the polarization effect and PCD of transformation ability of emergency scientific research achievements in different regions under major public health emergencies are analyzed. The study finds that:

1. In the static evaluation of transformation ability of the emergency scientific research results of different scientific research subjects under the “COVID-19” epidemic, the average value of the transformation ability of the emergency results (from March 2020 to May 2021) is ranked as enterprise, institution, individual, university, and research institute. In the dynamic evaluation of each subject's transformation ability of the emergency scientific research results, enterprise has the strongest ability to transform emergency scientific research results, which exceeds the average value. In addition, enterprise ranks high in all aspects of the transformation of emergency achievements, and the advantage of patent maintenance period is more prominent; other subjects have smaller differences in the number of valid invention patents and claims, and the gap between their patent maintenance period and enterprises is larger.
2. In the static evaluation of the transformation ability of emergency science research achievements in different regions, the top 5 regions in terms of the average value of transformation ability are Guangdong, Beijing, Jiangsu, Shanghai, and Tianjin. In the dynamic evaluation of the transformation ability of emergency scientific research results in each region, Guangdong has the strongest transformation ability of emergency scientific research results, which exceeds the average value. In addition, Guangdong ranks first in the dynamic evaluation of all indicators of emergency achievements transformation ability, with more prominent advantages in patent maintenance period and number of claims; Beijing ranks first in the dynamic evaluation of the number of valid invention patents; Jiangsu, Shanghai, and Tianjin are more consistent in the dynamic evaluation of all indicators, and Jiangsu has certain advantages in the patent maintenance period.
3. During the response to the “COVID-19” epidemic, the top 3 comprehensive economic zones in terms of dynamic evaluation of the transformation capacity of emergency scientific research results are: Eastern Coastal Economic Zone, Northern Coastal Economic Zone, and Southern Coastal Economic Zone, with the strong transformation capacity of emergency scientific research results; the dynamic evaluation values of transformation ability of emergency scientific research achievement in Middle Yellow River Economic Zone and Northwest Economic Zone are low, and the transformation ability is weak. In the process of epidemic response, the eight comprehensive economic zones have significant differences in the transformation ability of emergency scientific research results and unbalanced spatial distribution.
4. The polarization degree of transformation capability of emergency science research results is measured and analyzed for the whole country and eight comprehensive economic zones. Firstly, the SPDs of transformation capability of emergency scientific research results in China fluctuates during the response to the “COVID-19” epidemic, and the polarization level is low, indicating that the resource gathering status of national emergency research is constantly adjusting with the epidemic development stage, and the resource aggregation process in the global scope has not yet shown the characteristics of order and large scale. The “polarization” and “diffusion” of transformation capability of emergency scientific research results in China are alternating, and the polarization effect is weak; the dynamic polarization level of transformation ability of emergency scientific research results in China is low, indicating that the transformation ability of emergency scientific research results at the nationwide level does not form a significant polarization effect under the consideration of the influence of time factors. Secondly, the static polarization level of transformation ability of emergency scientific research results in the Northern Coastal Economic Zone, Eastern Coastal Economic Zone, and Southern Coastal Economic Zone in each month differ significantly, and the dynamic polarization degree is low; the transformation ability of emergency scientific research results has not formed a more obvious and stable polarization effect, and under the “COVID-19” epidemic, their resources gathering of emergency scientific research results transformation has not formed an orderly and large-scale development trend. Third, within the Northern Coastal Economic Zone, Tianjin has the largest PCD of transformation capability of emergency scientific research results; the PCDs of Tianjin, Hebei, and Shandong are all greater than 0, which promote the polarization effect of transformation capacity of emergency scientific research results in the Northern Coastal Economic Zone. The PCD of Beijing is less than 0, and it has an inhibiting effect on the polarization effect of emergency research results transformation capacity in the Northern Coastal Economic Zone. Within the Eastern Coastal Economic Zone, the PCD of emergency scientific research results transformation capacity in Shanghai is the largest; the PCDs of Shanghai, Jiangsu, and Zhejiang are all greater than 0, which all have a positive contribution to the polarization effect of transformation capacity of emergency scientific research results in the Eastern Coastal Economic Zone. Within the Southern Coastal Economic Zone, Guangdong has the largest PCD of emergency scientific research results transformation ability; the PCDs of Fujian, Guangdong, and Hainan are all greater than 0, which all promote the polarization effect of transformation ability of emergency scientific research results in the Southern Coastal Economic Zone.

It should be noted that there are also limitations in this paper. In the context of COVID-19, the statistical caliber and focus of progress data related to emergency scientific research result transformation within nationwide are inconsistent, which limits the availability of evaluation index data and affects the diversification of evaluation indicators. In the follow-up study, relevant data can be further collected and organized, and relevant achievements information of emergency scientific research projects can be supplemented, so as to improve the evaluation indexes of the transformation capability of emergency scientific research achievements under public health emergencies. In addition, considering the strong innovation strength and R&D potential possessed by enterprises, we can focus on the transformation of enterprise's emergency scientific research results under major public health emergencies and further analyze the spatial-temporal evolution characteristics of emergency scientific research results transformation ability, the transformation efficiency of emergency science research results, and emergency scientific research resources allocation.

## 6. Innovations

The innovations of this work are reflected in the following aspects. (1) The innovation of the evaluation method. Considering the lack of data directly related to major public emergencies, the statistical cycles and calibers of different regions are different, and the data vary greatly in different regions and different periods; neither the singly subjective weighting method nor objective weighting method is suitable for the evaluation of the transformation ability of emergency scientific research achievements. Therefore, an improved minimum distance-maximum entropy combination weight method is proposed to evaluate the transformation capacity of emergency scientific research results under public health emergencies, so as to improve the rationality, accuracy, and credibility of evaluation results. (2) The innovation of the evaluation index system. The major public emergencies have a huge impact on the transformation of emergency scientific research results and bring complex consequences. It is necessary to combine the characteristics of scientific research results transformation in the context of public emergencies, and comprehensively select evaluation indicators to construct a comprehensive evaluation index system of transformation ability for emergency scientific research achievements under the background of major public emergencies. (3) This paper uses progress data (monthly) to realize the timely evaluation of transformation capability for emergency scientific research achievements. Different from most existing literature that uses annual data, the use of monthly progress data for analysis is more conducive to obtaining the immediate characteristics of achievements transformation capability under the impact of emergencies, and provides a reliable basis for efficient, accurate, and timely decision-making. (4) The ER index and the PCD are further improved. This will enrich the research methods of the spatial effect of the transformation capacity of emergency scientific research achievements and provide a reliable analysis tool for the subsequent study of the transformation capacity of emergency scientific research achievements.

## Figures and Tables

**Figure 1:** The logical frame structure diagram.

**Figure 2:** Static evaluation results of the transformation ability of emergency scientific research achievements (subject difference perspective).

**Figure 3:** Dynamic evaluation results of first-level indicators (subject difference perspective).

**Figure 4:** Static evaluation results of the transformation ability of emergency scientific research achievements (region difference perspective).

**Figure 5:** Dynamic evaluation results of first-level indicators (region difference perspective).

**Figure 6:** The static evaluation of transformation ability of emergency scientific research achievements in the 8 comprehensive economic zones.

**Figure 7:** Polarization degree of transformation ability of emergency scientific research achievements (nationwide).

**Figure 8:** Static polarization degree of transformation ability of emergency scientific research achievements (part of comprehensive economic zones).

**Table 1:** The assignment reference of *r*_*k*_.

*r*_*k*_	Interpretation
1.000	Indexes *x*_(*k* − 1)_ and *x*_*k*_ are equally important
1.200	Index *x*_(*k* − 1)_ is slightly more important(than *x*_*k*_)
1.400	Index *x*_(*k* − 1)_ is more important(than *x*_*k*_)
1.600	Index *x*_(*k* − 1)_ is strongly more important(than *x*_*k*_)
1.800	Index *x*_(*k* − 1)_ is seriously more important(than *x*_*k*_)

**Table 2:** The importance of time.

*θ*	Interpretation
0.100	Great attention to recent data
0.300	Attention to recent data
0.500	Equal attention to data from all periods
0.700	Attention to long-term data
0.900	Great importance to long-term data
0.200, 0.400, 0.600, 0.800	Corresponding to the intermediate situation of the above two adjacent judgments

**Table 3:** Evaluation index.

Index name	Index symbol	Index attribute	Index interpretation
Number of valid invention patents	*X*1	+	The number of patents approved and granted by the SIPO. It is not only a key indicator of patent quality but also an important indicator of industrial economic employment contribution. A valid invention patent is more conducive to obtaining the competitive advantage in technology and product innovation.

Patent maintenance period	*X*2	+/−	It is one of the critical indicators to reflect the effectiveness of patent system and the merits of patent maintenance system, which is seen as a key factor in measuring the value of technology and economics for the patent. The longer the patent maintenance period, the higher the innovation quality, competitive strength, and economic value of the patented technology, that is, the more likely the patented technology to create economic benefits for the patent holder. At the same time, the cost of patent maintenance should be considered and the maintenance period should be set rationally.

Number of patent claims	*X*3	+	It is the core of the patent, and determines the scope of patent protection. The more claims a patent has, the more key features of the patented technology, and the more cutting-edge, important, and economically valuable the patent is.

**Table 4:** Improved combination evaluation weight (subject difference perspective).

Index symbol	202003	202004	202005	202006	……	202102	202103	202104	202105
*X*1	0.355	0.369	0.342	0.310	……	0.321	0.323	0.325	0.337
*X*2	0.319	0.354	0.367	0.352	……	0.388	0.381	0.386	0.372
*X*3	0.325	0.277	0.290	0.338	……	0.291	0.295	0.289	0.290

**Table 5:** Static evaluation results of the transformation ability of emergency scientific research achievements (subject difference perspective).

Subject	202003	202004	202005	……	202102	202103	202104	202105	Mean	Rank
Enterprise	0.584	0.999	0.999	……	0.950	0.920	0.980	0.999	0.920	1
Institution	0.674	0.235	0.254	……	0.197	0.160	0.337	0.326	0.256	2
Individual	0.692	0.122	0.097	……	0.089	0.051	0.099	0.158	0.158	3
University	0.007	0.003	0.251	……	0.184	0.089	0.127	0.161	0.152	4
Research institute	0.007	0.003	0.083	……	0.196	0.113	0.189	0.004	0.126	5

**Table 6:** The time series weights.

Month	2020.03	2020.04	2020.05	2020.06	……	2021.02	2021.03	2021.04	2021.05
*w*_*t*_	0.037	0.040	0.043	0.046	……	0.086	0.093	0.100	0.108

**Table 7:** Dynamic evaluation results of the transformation ability of emergency scientific research achievements (subject difference perspective).

Subject	Enterprise	Institution	Individual	University	Research institute	Mean
*L*_*j*_	0.933	0.251	0.141	0.156	0.134	0.333
Rank	1	2	4	3	5	

**Table 8:** Dynamic evaluation results of first-level indicators (subject difference perspective).

Index symbol	Enterprise	Institution	Individual	University	Research institute	Mean
*X*1	0.311 (1)	0.136 (2)	0.071 (4)	0.074 (3)	0.066 (5)	0.135
*X*2	0.342 (1)	0.017 (2)	0.003 (4)	0.003 (3)	0.003 (5)	0.077
*X*3	0.280 (1)	0.098 (2)	0.067 (4)	0.079 (3)	0.065 (5)	0.121

**Table 9:** Improved combination evaluation weight (region difference perspective).

Index symbol	202003	202004	202005	202006	……	202102	202103	202104	202105
*X*1	0.509	0.414	0.434	0.456	……	0.395	0.474	0.407	0.486
*X*2	0.193	0.236	0.189	0.187	……	0.179	0.155	0.131	0.154
*X*3	0.298	0.350	0.378	0.357	……	0.426	0.371	0.462	0.360

**Table 10:** Static evaluation results of the transformation ability of emergency scientific research achievements (region difference perspective).

Region	202003	202004	202005	202006	……	202102	202103	202104	202105	Mean	Rank
Beijing	0.004	0.244	0.298	0.465		1.000	0.558	0.872	0.874	0.580	2
Tianjin	0.004	0.003	0.091	0.167		0.132	0.001	0.001	0.004	0.180	5
……	……	……	……	……	……	……	……	……	……	……	
Liaoning	0.702	0.003	0.001	0.001		0.017	0.001	0.001	0.198	0.067	10
……	……	……	……	……	……	……	……	……	……	……	
Shanghai	0.004	0.003	0.253	0.274		0.052	0.182	0.191	0.750	0.272	4
Jiangsu	0.714	0.117	0.237	0.111		0.197	1.000	0.541	0.500	0.541	3
Zhejiang	0.004	0.003	0.001	0.001		0.174	0.076	0.257	0.004	0.096	9
Anhui	0.814	0.003	0.001	0.001		0.001	0.001	0.038	0.126	0.098	8
Fujian	0.004	0.003	0.001	0.001		0.001	0.076	0.001	0.004	0.051	15
……	……	……	……	……	……	……	……	……	……	……	
Shandong	0.004	0.003	0.087	0.001		0.042	0.068	0.206	0.004	0.062	12
……	……	……	……	……	……	……	……	……	……	……	
Hubei	0.004	0.072	0.075	0.001		0.049	0.119	0.067	0.181	0.065	11
Hunan	0.004	0.269	0.091	0.119		0.056	0.001	0.001	0.004	0.101	7
……	……	……	……	……	……	……	……	……	……	……	
Guangdong	0.004	1.000	1.000	1.000		0.439	0.382	0.832	0.592	0.673	1
Guangxi	0.004	0.003	0.079	0.001		0.001	0.001	0.169	0.004	0.051	14
……	……	……	……	……	……	……	……	……	……	……	
Sichuan	0.004	0.003	0.001	0.062		0.235	0.283	0.001	0.346	0.136	6
……	……	……	……	……	……	……	……	……	……	……	
Ningxia	0.004	0.003	0.001	0.001		0.001	0.001	0.366	0.172	0.054	13
……	……	……	……	……	……	……	……	……	……	……	

Mean	0.076	0.067	0.078	0.075		0.083	0.100	0.128	0.129		

**Table 11:** Dynamic evaluation results of the transformation ability of emergency scientific research achievements (region difference perspective).

Region	*L*_*j*_	Rank
Beijing	0.651	2
Tianjin	0.178	5
Hebei	0.050	17
Shanxi	0.022	21
Inner Mongolia	0.002	27
Liaoning	0.055	13
Jilin	0.037	19
Heilongjiang	0.013	22
Shanghai	0.288	4
Jiangsu	0.567	3
Zhejiang	0.113	7
Anhui	0.082	9
Fujian	0.050	16
Jiangxi	0.002	27
Shandong	0.067	12
Henan	0.054	14
Hubei	0.071	11
Hunan	0.087	8
Guangdong	0.654	1
Guangxi	0.051	15
Hainan	0.002	27
Chongqing	0.006	25
Sichuan	0.157	6
Guizhou	0.031	20
Yunnan	0.042	18
Tibet	0.002	27
Shaanxi	0.008	23
Gansu	0.007	24
Qinghai	0.002	27
Ningxia	0.075	10
Xinjiang	0.005	26

**Table 12:** Dynamic evaluation results of first-level indicators (region difference perspective).

Index symbol	Beijing	Tianjin	Shanghai	Jiangsu	Guangdong	Mean
*X*1	0.346 (1)	0.099 (5)	0.149 (4)	0.283 (3)	0.308 (2)	0.237
*X*2	0.055 (2)	0.002 (5)	0.005 (4)	0.051 (3)	0.064 (1)	0.035
*X*3	0.250 (2)	0.077 (5)	0.134 (4)	0.233 (3)	0.283 (1)	0.195

**Table 13:** Transformation ability of emergency scientific research achievements in the eight comprehensive economic zones.

Comprehensive economic zones	202003	202004	202005	202006	202007	202008	202009	202010	202011	202012	202101	202102	202103	202104	202105	Dynamic evaluation	Rank
Northeast economic region	0.237	0.003	0.001	0.017	0.001	0.052	0.002	0.062	0.054	0.086	0.002	0.006	0.001	0.001	0.068	0.035	6
Northern coastal economic zone	0.004	0.063	0.139	0.158	0.095	0.314	0.145	0.414	0.173	0.413	0.317	0.305	0.190	0.290	0.221	0.237	2
Eastern coastal economic zone	0.241	0.041	0.164	0.129	0.372	0.320	0.450	0.534	0.150	0.471	0.364	0.141	0.419	0.329	0.418	0.322	1
Southern coastal economic zone	0.004	0.335	0.334	0.334	0.367	0.229	0.108	0.395	0.334	0.271	0.137	0.147	0.153	0.278	0.200	0.235	3
Middle yellow river economic zone	0.004	0.029	0.001	0.015	0.001	0.002	0.002	0.002	0.001	0.054	0.025	0.001	0.048	0.034	0.048	0.022	7
Middle yangtze river economic zone	0.207	0.087	0.042	0.030	0.082	0.108	0.022	0.065	0.020	0.103	0.072	0.027	0.031	0.027	0.078	0.061	4
Southwest economic zone	0.004	0.044	0.039	0.013	0.043	0.114	0.050	0.103	0.027	0.071	0.032	0.066	0.058	0.071	0.072	0.058	5
Northwest economic zone	0.004	0.003	0.001	0.001	0.022	0.002	0.002	0.002	0.001	0.051	0.002	0.008	0.001	0.074	0.037	0.018	8

**Table 14:** Polarization degree of transformation ability of emergency scientific research achievements (part of comprehensive economic zones).

Comprehensive economic zones	Static polarization degree																	Dynamic polarization degree
	202003	202004	202005	202006	202007	202008	202009	202010	202011	202012	202101	202103	202104	202105	Mean	Min	Max	
Northern coastal Economic zone	≤0.001	≤0.001	0.392	0.147	0.141	0.123	0.164	0.112	0.261	0.145	0.079	0.180	0.135	≤0.001	0.132	≤0.001	0.392	0.128
Eastern coastal economic zone	≤0.001	≤0.001	0.031	0.283	0.155	0.120	0.125	0.071	0.404	0.101	0.121	0.130	0.203	0.083	0.133	≤0.001	0.404	0.141
Southern coastal economic zone	≤0.001	≤0.001	≤0.001	≤0.001	0.050	≤0.001	≤0.001	0.083	≤0.001	≤0.001	0.240	0.177	≤0.001	≤0.001	0.037	≤0.001	0.240	0.043

**Table 15:** Polarization contribution degree of transformation ability of emergency scientific research achievements (part of comprehensive economic zones).

Region	Polarization contribution degree	Rank
Northern coastal economic zone		
Beijing	−0.597	4
Tianjin	0.344	1
Hebei	0.179	2
Shandong	0.176	3

Eastern coastal economic zone		
Shanghai	0.483	1
Jiangsu	0.223	2
Zhejiang	0.065	3

Southern coastal economic zone		
Fujian	0.206	2
Guangdong	0.612	1
Hainan	0.030	3

## Data Availability

The datasets generated during and/or analyzed during the current study are available from the corresponding author on reasonable request.
